The article "Ubiquitin ligase SMURF1 functions as a prognostic marker and promotes growth and metastasis of clear cell renal cell carcinoma" was retracted in 2022. Reasons: duplicated images; signs of a paper mill; unreliable results or conclusions.

# Ubiquitin ligase SMURF1 functions as a prognostic marker and promotes growth and metastasis of clear cell renal cell carcinoma

**DOI:** 10.1002/2211-5463.12204

**Published:** 2017-02-23

**Authors:** Mang Ke, Licai Mo, Weilin Li, Xianjun Zhang, Feiping Li, Hongyuan Yu

**Affiliations:** ^1^ Department of UrologyTaizhou Hospital of Zhejiang ProvinceWenzhou Medical UniversityLinhaiZhejiang ProvinceChina

**Keywords:** ccRCC, DAB2IP, metastasis, proliferation, signaling pathway, SMURF1

## Abstract

Smad ubiquitin regulatory factor 1 (SMURF1), a recently identified E3 ubiquitin ligase, targets substrate proteins for ubiquitination and proteasomal degradation. Previous studies have reported that SMURF1 also functions as an oncogene in human cancers. However, the clinical value of SMURF1 and its role in clear cell renal cell carcinoma (ccRCC) are unknown. SMURF1 expression was analyzed in 100 cases of ccRCC and matched tumor‐adjacent specimens. SMURF1 was prominently overexpressed in ccRCC specimens compared with tumor‐adjacent specimens. Increased levels of SMURF1 were also observed in ccRCC cell lines. Clinicopathological detection verified that SMURF1 expression was associated with advanced tumor node metastasis stage, large tumor size and vascular invasion of ccRCC patients. Moreover, Kaplan–Meier analysis found that SMURF1 elevation led to adverse overall survival and disease‐free survival. Multivariate Cox regression analysis revealed that SMURF1 expression was an independent marker for prognosis prediction. Further experiments illustrated that SMURF1 knockdown significantly inhibited growth and metastasis of 769P cells, while SMURF1 overexpression promoted proliferation, migration and invasion in OSRC‐2 cells. Mechanistically, SMURF1 inversely regulated the expression of DAB2 interacting protein, which negatively mediated the activation of both the ERK/RSK1 and PI3K/AKT/mTOR pathways in ccRCC cells. Taken together, these results suggest that SMURF1 might be a promising biomarker and target for novel treatment of human ccRCC.

**Abbreviations**
ccRCC: clear cell renal cell carcinoma
DAP2IP: DAB2 interacting protein
ERK: extracellular signal‐regulated kinase
GAPDH: glyceraldehyde 3‐phosphate dehydrogenase
IHC: immunohistochemistry
mTOR: mechanistic target of rapamycin
MTT: 3‐(4,5‐dimethylthiazol‐2‐yl)‐2,5‐diphenyl‐tetrazolium bromide
PI3K: phosphoinositide 3‐kinase
qRT‐PCR: quantitative real‐time polymerase chain reaction
RCC: renal cell carcinoma
RSK1: ribosomal S6 kinase 1
shRNA: small hairpin RNA
SMURF1: Smad ubiquitin regulatory factor 1
TNM: tumor node metastasis

Renal cell carcinoma (RCC) represents one of the commonest malignancies characterized by an adverse clinical outcome 1. Approximately 75% of RCC patients have the clear cell renal cell carcinoma subtype (ccRCC) 2. Radical surgery might be the only hope for curing RCC in the stage of precursor lesions 3. However, even after surgical resection, radiotherapy and chemotherapy provide little benefit 4. Previous studies have identified that a few molecular markers were correlated with prognosis, but the mechanism of RCC is still unqualified 5. Therefore, there is an urgent need to identify an oncogenesis‐associated biomarker that would be helpful for developing novel treatments for RCC.

The article "Ubiquitin ligase SMURF1 functions as a prognostic marker and promotes growth and metastasis of clear cell renal cell carcinoma" was retracted in 2022. Reasons: duplicated images; signs of a paper mill; unreliable results or conclusions.

Smad ubiquitin regulatory factor 1 (SMURF1), a recently identified E3 ubiquitin ligase, targets substrate proteins for ubiquitination and proteasomal degradation 6. Increasing evidence has shown that SMURF1 exerts a promoting effect in carcinogenesis by targeting downstream proteins for proteolysis. Epidermal growth factor‐induced SMURF1 overexpression promotes breast cancer cell migration and invasion by targeting RhoA 7. Tumor necrosis factor receptor‐associated factor 4 is also reported to be a substrate protein of SMURF1 and promotes migration of breast cancer cells 8. SMURF1 was identified as a potential oncogene and good candidate for therapeutic target of pancreatic cancer 9, 10. The overexpression of SMURF1 is observed in human colorectal cancer, and contributes to tumor progression and poor prognosis 11. Several studies have reported the upstream regulator of SMURF1, IQ motif containing GTPase activating protein 1, promotes the ubiquitination and degradation of transforming growth factor β receptor II by facilitating the targeting of SMURF1 to the plasma membrane in hepatic stellate cells 12. Casein kinase‐2 interacting protein‐1 suppresses colon cancer cell growth and migration by inhibiting SMURF1 synthesis and facilitating SMURF1 autodegradation 13. Furthermore, SMURF1 is recognized as a direct target of miR‐497 in ovarian cancer cells and acts as a pro‐metastatic factor 14. But, the clinical significance of SMURF1 and its role in human ccRCC remain poorly investigated.

This study showed that elevation of SMURF1 expression predicted poorer survival. We also showed that SMURF1 promoted ccRCC cell growth and metastasis *in vitro*. Notably, SMURF1 regulated the expression of DAB2 interacting protein (DAP2IP) as well as the activation of the extracellular signal‐regulated kinase (ERK)/ribosomal S6 kinase 1 (RSK1) and phosphoinositide 3‐kinase (PI3K)/AKT/mechanistic target of rapamycin (mTOR) pathways. In conclusion, this work provided the first evidence that SMURF1 was a significant biomarker and a potential target for ccRCC.

## Materials and methods

### Patients

One hundred cases of ccRCC and matched tumor‐adjacent specimens were obtained from the Department of Urology, Taizhou Hospital of Zhejiang Province, Wenzhou Medical University between January 2009 and December 2011, with a median follow‐up time of 37.4 months. Tissue specimens were conserved in liquid nitrogen for quantitative real‐time PCR (qRT‐PCR) and 10% formalin for immunohistochemistry (IHC) until use. Informed consent for all samples was obtained before use. All cases were primary ccRCC and were reviewed by a pathologist. Tumor grade was assessed according to the Fuhrman nuclear grade 15. Clinicopathological information for the patients is represented in Table 1. ccRCC was localized in 89 patients, and 11 patients had distant metastases at the time of diagnosis. Metastasis occurred in 12 cases of ccRCC patients during follow‐up and 38 patients had died at last follow‐up. The metastasized patients received sunitinib. The Ethics Committee of Wenzhou Medical University approved this study according to the Declaration of Helsinki.

The article "Ubiquitin ligase SMURF1 functions as a prognostic marker and promotes growth and metastasis of clear cell renal cell carcinoma" was retracted in 2022. Reasons: duplicated images; signs of a paper mill; unreliable results or conclusions.

**Table 1:** The correlation between SMURF1 and clinicopathological features in clear cell renal cell carcinoma patients. TNM, tumor node metastasis

Characteristic	Total	SMURF1 expression		*P*
		Positive (67)	Negative (33)	
Age				
< 60 years	44	31	13	0.515
≥ 60 years	56	36	20	
Gender				
Male	64	45	19	0.348
Female	36	22	14	
TNM stage				
I + II	79	49	30	0.040^a^
III + IV	21	18	3	
G grade				
G1 + G2	81	51	30	0.076
G3	19	16	3	
Vascular invasion				
Positive	82	51	31	0.029^a^
Negative	18	16	2	
Tumor size				
< 5 cm	61	36	25	0.034^a^
≥ 5 cm	39	31	8	

a Statistically significant.

### Cell culture and transfection

ccRCC‐derived cell lines (769P and OSRC‐2) and a normal renal cell line (HK2) were obtained from the Cell Bank of Shanghai Institute of Cell Biology (Chinese Academy of Medical Science, Shanghai, China). Cell lines were cultured in DMEM with 10% fetal bovine serum (Gibco/Thermo Fisher Scientific, Waltham, MA, USA) with antibiotics (Sigma‐Aldrich, St. Louis, MO, USA) in an incubator containing a 5% CO_2_ humidified atmosphere at 37 °C.

Small hairpin RNA (shRNA) targeting SMURF1 and non‐targeting (NT) shRNA were obtained from Santa Cruz Biotechnology (Dallas, TX, USA). shRNA vectors were transferred into cells using lipofectamine 2000 (Thermo Fisher Scientific) on the basis of the manufacturer's recommendation. Retroviral vector pMMP‐SMURF1 was generated by inserting the cDNA into pMMP. Retrovirus packaging and transduction were described previously 16.

### Immunohistochemistry

The tissues that were previously formalin‐fixed and paraffin‐embedded were sliced into 4 μm sections, and underwent deparaffination and then rehydration. Antigen retrieval, suppression of endogenous peroxidase activity and 10% skim milk blocking were performed before primary antibody incubation. SMURF1 (Abcam, Cambridge, MA, USA) antibody was used as primary antibody overnight at 4 °C. The slides were subsequently incubated with peroxidase conjugated secondary antibody (ZSGB Bio, Beijing, China) for 90 min, and a solution of peroxidase‐labeled polymer, 2,4‐diaminobutyric acid, was used for signal development for 5 min. The sections were counterstained with hematoxylin followed by dehydrating and mounting. Staining intensity was scored manually by two independent experienced pathologists as follows: no staining = 0, weak staining = 1, moderate staining = 2 and strong staining = 3.

The article "Ubiquitin ligase SMURF1 functions as a prognostic marker and promotes growth and metastasis of clear cell renal cell carcinoma" was retracted in 2022. Reasons: duplicated images; signs of a paper mill; unreliable results or conclusions.

### Quantitative real‐time PCR

Total RNA was drawn using Trizol (Invitrogen/Thermo Fisher Scientific) from fresh‐frozen tissues. cDNAs were synthesized from 2 μg total RNA using TIANScript RT Kit (Tiangen Biotech, Beijing, China). Quantitative real‐time PCR was performed using the SYBR Green PCR Master Mix (Toyobo, Osaka, Japan) in a final volume of 10 μL in an ABI 7300 Fast PCR machine (Applied Biosystems, Foster City, CA, USA). Glyceraldehyde 3‐phosphate dehydrogenase (GAPDH) was employed as a reference gene to normalize the expression of SMURF1 mRNA. Data are presented as relative quantification based on the calculation of $2^{-\Delta C_{t}}$. Δ*C*_t_ was derived from subtracting the *C*_t_ value of reference cDNA from the *C*_t_ value of the cDNA of interest. The primers used for target genes were purchased from Sangon Biotech (Shanghai, China). Primer sequences were as follows: SMURF1 forward, 5′‐CTA CCA GCG TTT GGA TCT AT‐3′; reverse, 5′‐TGT CTC GGG TCT GTA AAC T‐3′. GAPDH forward, 5′‐CAA GCT CAT TTC CTG GTA TGA C‐3′; reverse, 5′‐CAG TGA GGG TCT CTC TCT TCC T‐3′.

### Proliferation assay

Cells after transfection were gathered for cell growth assay (3‐(4,5‐dimethylthiazol‐2‐yl)‐2,5‐diphenyl‐tetrazolium bromide (MTT) assay) following the manufacturer's recommendation (Roche, Indianapolis, IN, USA). In summary, cells were grown in 96‐well plates containing 100 μL DMEM per well. After transfection for 24, 48, 72 and 96 h, respectively, 10 μL of MTT was added to each well; after incubation for 4 h the medium was undocked and subsequently 150 μL DMSO was added per well. The results represent the average of three independent replicates. For the colony formation assay, 2000 ccRCC cells were cultured on six‐well plates, and 14–21 days after seeding, cell colonies stained with crystal violet and counted.

### Wound healing assay

ccRCC cells transduced with corresponding vectors were seeded in six‐well plates to form a single confluent cell layer. A wound was made with 100 μL pipette tip in the confluent cell layer; 0 and 24 h after wound scratching, the width of the wound was photographed with a phase‐contrast microscope.

The article "Ubiquitin ligase SMURF1 functions as a prognostic marker and promotes growth and metastasis of clear cell renal cell carcinoma" was retracted in 2022. Reasons: duplicated images; signs of a paper mill; unreliable results or conclusions.

### Transwell invasion assay

We determined the cell invasion capacities by using Transwell chambers of pore size 8 μm (Coring Costar, Cambridge, MA, USA). Twenty‐four hours after transduction, 5 × 10^4^ cells were cultured in the 1 : 9 diluted Matrigel‐coated (BD Biosciences, Franklin Lakes, NJ, USA) upper chamber with 250 μL serum‐free DMEM, and 700 μL DMEM with 10% fetal bovine serum was added in the lower chamber. After 24 h, the cells were fixed with paraformaldehyde and those in upper chamber were removed. Cells in the lower chamber were subsequently stained using 0.1% crystal violet solution and photographed.

### Western blotting

Cancer cells were dissociated in RIPA lysis buffer (P0013D) (Beyotime, Haimen, China) and PMSF (ST506) (Beyotime). Split products were centrifuged at 18 500 ***g***, and the supernatants were collected. A Bradford Protein Assay Kit (P0006) (Beyotime) was used to analyze protein concentration, and the proteins were subject to 10% SDS/PAGE electrophoresis. After separation the proteins were transferred onto poly(vinylidene difluoride) membranes (Sigma‐Aldrich), and the membranes were blocked with 5% skim milk (Guangming, Shanghai, China) and incubated with primary antibody at 4 °C overnight. Then, specimens were hatched with secondary antibody conjugated with horseradish peroxidase (Cell Signaling Technology, Beverly, MA, USA). Signals were detected using a horseradish peroxidase chemiluminescent kit (Thermo Fisher Scientific) using an optional CCD camera and image processing system (Bio‐Rad, Hercules, CA, USA). GAPDH (G8140, US Biological, Swampscott, MA, USA) was used as a loading control. SMURF1, DAB2IP and p‐RSK1 (Ser380) were purchased from Abcam. p‐AKT (Ser473), AKT, p‐mTOR (Ser2448), mTOR, p‐ERK (Thr202/Tyr204), ERK and RSK1 were obtained from Cell Signaling Technology.

### Statistical analysis

Data were presented as the mean ± SEM and analyzed by prism 5 software (GraphPad Software, Inc., San Diego, CA, USA) and spss version 13 (SPSS, Chicago, IL, USA). The chi‐squared test was employed to explore the association between two variables. Student's *t* test and ANOVA were carried out to analyze continuous variables. Survival curves were constructed and differences among groups were calculated using the Kaplan–Meier method and log‐rank test. The multivariate Cox regression analysis was performed to reveal the prognostic significance of SMURF1 expression. The value of *P* < 0.05 was considered to have statistical significance.

The article "Ubiquitin ligase SMURF1 functions as a prognostic marker and promotes growth and metastasis of clear cell renal cell carcinoma" was retracted in 2022. Reasons: duplicated images; signs of a paper mill; unreliable results or conclusions.

## Results

### SMURF1 is overexpressed in ccRCC

One hundred samples of ccRCC and matched tumor‐adjacent specimens were detected by immunohistochemistry for SMURF1 staining. Sections with IHC score ≥ 1 were considered to show positive expression of SMURF1. Of the ccRCC tissues, 67% of the cases (score 1: 18 cases; score 2: 32 cases; score 3: 17 cases) showed positive staining of SMURF1, while SMURF1 signal was detected in only 35% (score 1: 15 cases; score 2: 16 cases; score 3: 4 cases) of samples of tumor‐adjacent specimens (*P* < 0.05, Fig. 1). Next, qRT‐PCR demonstrated that the level of SMURF1 mRNA in ccRCC tissues was up‐regulated compared with matched tumor‐adjacent specimens (*P* < 0.05, Fig. 2A). The expression of GAPDH mRNA was comparable in ccRCC and tumor‐adjacent tissues (Fig. S1). Moreover, the levels of SMURF1 expression in two ccRCC cell lines (769P and OSRC‐2) were significantly elevated over that in normal human renal cells (HK2) (*P* < 0.05, respectively, Fig. 2B). Thus, overexpression of SMURF1 potentiates an oncogenic role in ccRCC.

**Figure 1:** Immunohistochemistry of SMURF1 protein in clear cell renal cell carcinoma (ccRCC) and normal tissues. Representative immunohistochemical staining showing (A) normal kidney proximal tubular epithelium, and (B) weak, (C) moderate and (D) strong staining of ccRCC. Scale bar: 50 μm.

**Figure 2:** Expression differences and prognostic significance of SMURF1 in ccRCC. (A) Expression of SMURF1 mRNA in fresh‐frozen ccRCC tissues and matched tumor‐adjacent specimens. *n* = 50. (B) Relative expressions of SMURF1 mRNA in two ccRCC cell lines (769P and OSRC‐2) and normal human kidney cells (HK2). *n* = 3, *P < 0.05. (C,D) Based on the status of SMURF1 expression, SMURF1 positively expressing ccRCC patients had a notably decreased overall and disease‐free survival.

### Clinical significance of SMURF1 in ccRCC patients

To explore the clinical value of SMURF1, we correlated SMURF1 expression with clinical parameters of ccRCC patients. As shown in Table 1, patients with advanced tumor node metastasis (TNM) stage, vascular invasion and large tumor size showed a significantly higher positive rate of SMURF1 expression (*P* < 0.05, respectively). These results verify that elevation of SMURF1 expression may lead to ccRCC carcinogenesis. Notably, Kaplan–Meier analysis indicated SMURF1 positive expression significantly related to shortened overall and disease‐free survival in our specimens (*P* < 0.05, respectively, Fig. 2C,D). Furthermore, the multivariate Cox regression analysis revealed that SMURF1 expression was an independent marker for 5‐year overall and disease‐free survival (*P* < 0.05 for each, Table 2). Our data revealed that SMURF1 may act as a promising prognostic indicator for ccRCC patients.

The article "Ubiquitin ligase SMURF1 functions as a prognostic marker and promotes growth and metastasis of clear cell renal cell carcinoma" was retracted in 2022. Reasons: duplicated images; signs of a paper mill; unreliable results or conclusions.

**Table 2:** Multivariate Cox regression analysis of 5‐year overall and disease‐free survival of 100 clear cell renal cell carcinoma patients. HR, hazard ratio; TNM, tumor‐node‐metastasis

Variable	Overall survival			Disease‐free survival		
	HR	95% CI	*P*	HR	95% CI	*P*
Tumor size (≥ 5 cm *vs* < 5 cm)	1.90	0.73–4.98	0.189	2.34	0.95–5.81	0.066
Vascular invasion (Positive *vs* Negative)	1.68	1.00–2.85	0.051	1.59	0.89–2.85	0.118
TNM Stage (III + IV *vs* I + II)	3.06	1.52–6.16	0.002^a^	2.02	1.23–3.31	0.005^a^
SMURF1 expression (Positive *vs* Negative)	2.02	1.13–3.60	0.017^a^	2.19	1.14–4.20	0.024^a^

a Statistically significant.

### SMURF1 knockdown restrains ccRCC cell growth and metastasis

Because SMURF1 was overexpressed in ccRCC compared with normal, we speculated that the biological functions of SMURF1 may include participating in controlling cell growth and metastasis. To verify this hypothesis, SMURF1 expression was silenced by a specific shRNA in 769P cells (*P* < 0.05, Fig. 3A). MTT and colony formation assays were used to analyze the effect of SMURF1 on cell growth of ccRCC. We found that loss of SMURF1 restrained cell growth as compared with control in 769P cells (*P* < 0.05, Fig. 3B,C). All results support that SMURF1 is involved in ccRCC cell growth. To disclose the potential role of SMURF1 in the metastasis of ccRCC, we analyzed the migration and invasion of ccRCC cells using wound healing and transwell assays. The results suggested that SMURF1 knockdown caused a prominent reduction of migration and invasion of 769P cells as compared with control cells (*P* < 0.05, Fig. 3D,E). Taken together, the results prove that loss of SMURF1 can dramatically hold up ccRCC cell growth and metastasis *in vitro*.

**Figure 3:** Impact of SMURF1 knockdown on cell growth and metastasis. (A) 769P cells that were transduced with non‐targeting (NT) shRNA or SMURF1 shRNA were detected by western blotting for SMURF1 expression. *n* = 3, *P < 0.05. (B) MTT assays indicated that loss of SMURF1 prohibited proliferation in 769P cells. *n* = 3, *P < 0.05. (C) The relative number of colonies was reduced after SMURF1 silencing in 769P cells. *n* = 3, *P < 0.05. (D) Wound healing assays revealed that the migration of 769P cells was restrained by SMURF1 knockdown. (E) Transwell assays indicated that SMURF1knockdown reduced the number of invaded 769P cells. *n* = 3, *P < 0.05.

### SMURF1 overexpression leads to enhanced growth and metastasis of ccRCC cells

Next, OSRC‐2 cells were infected with empty vector (EV) and SMURF1 retroviruses. SMURF1 overexpression was confirmed by western blotting in OSRC‐2 cells (*P* < 0.05, Fig. 4A). Overexpression of SMURF1 notably enhanced the proliferation of OSRC‐2 cells (*P* < 0.05, Fig. 4B,C). Furthermore, wound healing assays indicated SMURF1 overexpression facilitated the migration of OSRC‐2 cells (Fig. 4D). In addition, SMURF1 overexpressing OSRC‐2 cells showed increased invasive ability compared with control cells (*P* < 0.05, Fig. 4E). Our data disclose that SMURF1 promotes the tumor growth and metastasis of ccRCC cells.

The article "Ubiquitin ligase SMURF1 functions as a prognostic marker and promotes growth and metastasis of clear cell renal cell carcinoma" was retracted in 2022. Reasons: duplicated images; signs of a paper mill; unreliable results or conclusions.

**Figure 4:** SMURF1 overexpression regulates cell growth and metastasis in OSRC‐2 cells. (A) OSRC‐2 cells that were infected with SMURF1 retroviruses or empty vector (EV) were tested by western blotting for SMURF1 expression. *n* = 3, *P < 0.05. (B) MTT assays revealed that SMURF1 overexpression facilitated proliferation in OSRC‐2 cells. *n* = 3, *P < 0.05. (C) The relative number of colonies was elevated after SMURF1 overexpression in OSRC‐2 cells. *n* = 3, *P < 0.05. (D) Wound healing assays demonstrated that the migration ability of OSRC‐2 cells was increased by SMURF1 overexpression. (E) SMURF1 overexpression promoted cell invasion in OSRC‐2 cells assessed by transwell assays. *n* = 3, *P < 0.05.

### The ERK/RSK1 and PI3K/AKT/mTOR signaling axis may be involved in the role of SMURF1

Previous research has identified that SMURF1 promotes cancer cell proliferation and migration by negatively regulating DAB2IP 17. Furthermore, DAB2IP knockdown leads to the activation of the ERK/RSK1 and PI3K/AKT/mTOR pathways in RCC cells 18. Thus, we explored whether the DAB2IP‐mediated ERK/RSK1 and PI3K/AKT/mTOR signaling axis was involved in the role of SMURF1 in ccRCC. Interestingly, we found that the expression of DAB2IP was increased and the levels of phosphorylated AKT, mTOR, ERK and RSK1 were remarkably decreased after SMURF1 knockdown in 769P cells. SMURF1 overexpression led to a decreased level of DAB2IP and increased activation of the ERK/RSK1 and PI3K/AKT/mTOR signaling pathways (Fig. 5). Therefore, these results indicated that the DAB2IP‐mediated ERK/RSK1 and PI3K/AKT/mTOR signaling axis might be involved in the function of SMURF1 in ccRCC cells.

**Figure 5:** SMURF1 regulates the activation of the ERK/RSK1 and PI3K/AKT/mTOR pathways by targeting DAB2IP in ccRCC cells. 769P and OSRC‐2 cells that were transfected with corresponding vectors (NT and SMURF1 shRNAs or EV and SMURF1 retroviruses) were subjected to immunoblotting for DAB2IP, p‐AKT, AKT, p‐mTOR, mTOR, p‐ERK, ERK, p‐RSK1 and RSK1. SMURF1 negatively regulated the expression of DAB2IP, and coordinately modulated the activation of the ERK/RSK1 and PI3K/AKT/mTOR pathways.

The article "Ubiquitin ligase SMURF1 functions as a prognostic marker and promotes growth and metastasis of clear cell renal cell carcinoma" was retracted in 2022. Reasons: duplicated images; signs of a paper mill; unreliable results or conclusions.

## Discussion

ccRCC is the most common subtype of RCC with increasing incidence, high metastatic potential and high mortality rate 19. Accumulating evidence has demonstrated that SMURF1 participates in many malignancies 7, 9, 10, 13, 14, 17. Dysregulation of SMURF1 is a common event found in various cancers including pancreatic cancer 9, 10, breast cancer 7, 8, ovarian cancer 14 and colorectal cancer 13. To the best of our knowledge, few articles in the literature have focused on the clinical value and role of SMURF1 in ccRCC up to now. Thus, further study of SMURF1 in ccRCC may be helpful in relation to this deadly disease. This work demonstrated the pattern of SMURF1 expression in ccRCC carcinogenesis and its potential prognostic significance in ccRCC patients, and further investigated its effect and mechanism in ccRCC cells.

The present study identified SMURF1 as a promising biomarker for prognosis of ccRCC patients. The expression of SMURF1 in ccRCC tissue was notably elevated compared with the tumor‐adjacent specimens, and its elevation correlated with advanced TNM stage, vascular invasion and large tumor size. Notably, multivariate Cox regression analysis revealed that SMURF1 expression was an independent marker for prognosis prediction. Additionally, we provided the first evidence that upregulation of SMURF1 in ccRCC was correlated with adverse outcome. Thus, SMURF1 potentially functions as a prognostic marker in ccRCC.

Then, we explored the biology of SMURF1 in ccRCC cells and showed that loss of SMURF1 expression could inhibit cell growth and metastasis *in vitro*. In turn, SMURF1 overexpression significantly promoted cell proliferation as well as migration and invasion in ccRCC cells. The prominent ability of SMURF1 to promote tumorigenesis supports that it plays an oncogenic role in ccRCC. Therefore, targeting SMURF1 may represent a favorable therapeutic strategy for ccRCC treatment. Next, we explored potential target genes participating step‐wise. We have shown that loss of SMURF1 up‐regulated DAB2IP expression and down‐regulated phosphorylated AKT, mTOR, ERK and RSK1. In contrast, SMURF1 overexpression reduced DAB2IP expression and enhanced the activation of the ERK/RSK1 and PI3K/AKT/mTOR signaling pathways in ccRCC cells. The expression of DAB2IP mRNA is regulated by DNA methylation in RCC, and DAB2IP CpG1 confers a poor survival of patients 20. Furthermore, DAB2IP has been previously identified as a tumor suppressor via restraining RCC cell growth and invasion by regulating the activation of the ERK/RSK1 and PI3K/AKT/mTOR pathways 21. The ERK/RSK1 pathway plays a critical role in determining the response of RCC cells to mTOR inhibitors via regulating hypoxia‐inducible factor 2α/p21 18. The mTOR pathway has been reported to be implicated in promoting RCC growth and metastasis 22. In addition, Yang *et al*. 23 revealed that infiltrating macrophages increase RCC cell invasion through induction of the epithelial–mesenchymal transition and increased cancer stem cell‐like populations via activation of AKT/mTOR signaling. Here, we provide a preliminary exploration showing that SMURF1 regulates the DAP2IP‐mediated ERK/RSK1 and PI3K/AKT/mTOR pathways, resulting in the induction of growth and metastasis in ccRCC cells.

The article "Ubiquitin ligase SMURF1 functions as a prognostic marker and promotes growth and metastasis of clear cell renal cell carcinoma" was retracted in 2022. Reasons: duplicated images; signs of a paper mill; unreliable results or conclusions.

In conclusion, we have provided the first evidence that SMURF1 has an oncogenic function important for ccRCC. Firstly, our results demonstrated that SMURF1 expression was elevated in ccRCC cell lines and tissues. Then, our clinical data suggested that SMURF1 may be used as a novel predictor for ccRCC. Moreover, SMURF1 overexpression in ccRCC cells not only resulted in growth and metastasis, but also increased the activation of the ERK/RSK1 and PI3K/AKT/mTOR pathways via DAB2IP inhibition. Taken together, our results verify that SMURF1 may serve as a potential target for cancer therapeutics of ccRCC.

## Conclusions

SMURF1 has been previously found to be implicated in cancer cell growth and metastasis, but its clinical value and biological function have remained poorly known in ccRCC. Here, we presented evidence that the level of SMURF1 in ccRCC tissues was notably elevated compared with normal specimens. Accordingly, the levels of SMURF1 were obviously up‐regulated in ccRCC cell lines compared with HK2 cells. The positive expression of SMURF1 was notably higher in patients with advanced TNM stage, vascular invasion and large tumor size. Importantly, survival analysis revealed that SMURF1 expression was an independent prognostic indicator for predicting overall and disease‐free survival of ccRCC patients. Knockdown of SMURF1 in 769P cells prominently inhibited growth and metastasis of cancer cells *in vitro*, while SMURF1 restoration had opposite effects on these behaviors in OSRC‐2 cells. Mechanically, SMURF1 exerted an oncogenic function by suppressing DAB2IP and subsequently enhanced the activation of the ERK/RSK1 and PI3K/AKT/mTOR pathways in ccRCC cells. Together this suggests that SMURF1 can potentially act as a prognostic predictor and a drug target for ccRCC patients.

## Author contributions

MK, LM, WL, XZ and FL carried out the cell biology and molecular biology experiments, participated in the sequence alignment and drafted the manuscript. MK and HY participated in the design of the study and performed the statistical analysis. HY conceived the study, and participated in its design and coordination and helped to draft the manuscript. All authors read and approved the final manuscript.

The article "Ubiquitin ligase SMURF1 functions as a prognostic marker and promotes growth and metastasis of clear cell renal cell carcinoma" was retracted in 2022. Reasons: duplicated images; signs of a paper mill; unreliable results or conclusions.

## Supporting information


**Fig. S1.** Expression of GAPDH mRNA in ccRCC and normal tissues.
